# Drug resistance of pathogens causing nosocomial infection in orthopedics from 2012 to 2017: a 6-year retrospective study

**DOI:** 10.1186/s13018-021-02234-7

**Published:** 2021-02-01

**Authors:** Xiaowei Yang, Runsheng Guo, Banglin Xie, Qi Lai, Jiaxiang Xu, Niya Hu, Lijun Wan, Min Dai, Bin Zhang

**Affiliations:** 1 Department of Orthopedics, First Affiliated Hospital of Nanchang University, No. 17 Yong Wai Zheng Street, Nanchang, 330006 Jiangxi China; 2 Department of Laboratory, First Affiliated Hospital of Nanchang University, No. 17 Yong Wai Zheng Street, Nanchang, 330006 Jiangxi China

**Keywords:** Hospital-acquired infections, Orthopedics, Drug resistance, Multidrug resistance

## Abstract

**Background:**

Hospital-acquired infections (HAIs) are an emerging global problem that increases in-hospital mortality, length of stay, and cost. We performed a 6-year retrospective study to provide valuable insight into appropriate antibiotic use in HAI cases. We also aimed to understand how hospitals could reduce pathogen drug resistance in a population that overuses antibiotics.

**Methods:**

All data (2012–2017) were obtained from the hospital information warehouse and clinical microbiology laboratory.

**Results:**

We isolated 1392 pathogen strains from patients admitted to the orthopedics department during 2012–2017. *Escherichia coli* (14.7%, 204/1392), *Enterobacter cloacae* (13.9%, 193/1392), and *Staphylococcus aureus* (11.3%, 157/1392) were the most common pathogens causing nosocomial infections. The dominant Gram-negative bacterium was *E. coli*, with high resistance to ampicillin, levofloxacin, cotrimoxazole, gentamicin, and ciprofloxacin, in that order. *E. coli* was least resistant to amikacin, cefoperazone-sulbactam. The most dominant Gram-positive bacterium was *S. aureus*, highly resistant to penicillin and ampicillin, but not resistant to fluoroquinolones and cotrimoxazole. Analysis of risk factors related to multidrug-resistant bacteria showed that patients with open fractures (Gustillo III B and IIIC) were significantly more susceptible to methicillin-resistant *S. aureus* infections (*p* < 0.05). Additionally, extended-spectrum β-lactamase-producing *E. coli* infections occurred significantly more often in patients with degenerative diseases (*p* < 0.05). Elderly patients tended to be more susceptible to multidrug-resistant bacterial infections, but this outcome was not statistically significant.

**Conclusions:**

Antimicrobial resistance is a serious problem in orthopedics. To effectively control antimicrobial resistance among pathogens, we advocate extensive and dynamic monitoring of MDR bacteria, coupled with careful use of antibiotics.

## Background

Hospital-acquired infections (HAIs), especially at surgical sites, are catastrophic complications that lead to higher in-hospital mortality, longer stay duration, and greater expense [1]. The USA alone spends over $33 billion on HAIs per year [2]. With the rapid development of invasive medical devices, HAI contributions to surgery-related morbidity and mortality have increased considerably [3]. This effect is particularly noticeable in orthopedics, an area that is very reliant on implants (e.g., internal fixation devices for bone fractures), wound dressings, and catheters. A 9-year retrospective study on 90551 patients who underwent elective spine surgery discovered that surgical site and urinary tract infection rates were 1.4% and 1.3%, respectively. Moreover, hospital stay duration was 1.48  ± 0.04 days longer and the cost was $8893  ± $148 greater for patients with HAIs [4]. Similarly, surgical site infections are the most common (25.2%) and the third most common (14.8%) reason for revision total knee arthroplasty and revision total hip arthroplasty, respectively [5].

Compounding HAI-related issues, antibiotic resistance among pathogens is a serious problem, owing to drug abuse stemming from hospital over-prescription as well as excessive self-medication in Chinese communities [6]. Furthermore, multidrug-resistant (MDR) bacteria have become increasingly prevalent, with notable examples being methicillin-resistant *Staphylococcus aureus* (MRSA) and extended-spectrum β-lactamase (ESBL)-positive *Escherichia coli* [7]. One study found that the MRSA isolation rate from patients ranges from 42.1 to 69.5% [8], which is very high despite a decreasing trend over 6 years. Likewise, another report isolated 30–40% MRSAs and 20–30% ESBL-positive *E. coli* [9]. The presence of MRSA or ESBL-positive *E. coli* in patients is associated with increased mortality [10, 11].

Most of the studies on pathogen resistance in orthopedics focused only on microbes causing surgical wound infections. However, HAIs are increasingly recognized as a major factor exacerbating such infections [12]. Therefore, this study aimed to understand resistance patterns of HAI-inducing microbes commonly found in orthopedics. Our findings should benefit efforts to encourage conservative antibiotic use when HAIs occur and to reduce pathogen drug resistance.

## Methods

### Location and study design

The department of orthopedics of the First Affiliated Hospital of Nanchang University has six wards and 350 beds, divided into seven sub-specialties: trauma, spine, joint, sports medicine, bone tumor and bone disease, and hand and foot microscopic repair and reconstruction, as well as pediatric orthopedics. Over 10,000 surgeries are performed annually, of which 60% are levels III and IV. Sickbed utilization rate is greater than 130%.

A retrospective surveillance study (2012–2017) was performed on nosocomial infections in orthopedics. Data were obtained from the hospital information warehouse and clinical microbiology laboratory. Nosocomial infections are defined as infections that begin when a patient is residing in a hospital, but were absent at the time of admission [13]. Here, we specifically classified infections as nosocomial if they occurred 48 h post-admission/post-surgery or later. Two researchers collected all relevant data, including basic patient information, bacteria strains cultivated, and antimicrobial resistance.

### Strain identification and antibiotic sensitivity testing

All clinical specimens, including wound secretions (skin and tissue that were already injured pre-surgery), incisional secretions (skin and tissue intact pre-surgery), urine, blood, and joint fluids, obtained from the orthopedics department between January 2012 and December 2017 were included in the analysis if they tested positive for pathogens. Identical strains from the same patient were excluded. Within 2 h of collection, specimens were stored in sterile culture tubes and sent to the microbiology laboratory. Different bacterial strains and antibacterial sensitivity were identified using the VITEK-2 automated system (bioMérieux Inc., France). Antimicrobial susceptibility was tested with the Kirby-Bauer method and minimum inhibitory concentrations, following updated guidelines from the Clinical and Laboratory Standards Institute [14]. *S. aureus* and *E. coli* were routinely tested with fourteen antibiotics, which are shown in Tables 2 and 3. *S. aureus* ATCC29213 and *E. coli* ATCC25922 strains were used in the antimicrobial susceptibility tests for quality control. Phenotypic confirmatory tests for extended-spectrum β-lactamase (ESBL)-producing *E. coli* and methicillin-resistant *S. aureus* (MRSA) were performed according to the latest CLSI guidelines [14].

### Statistical analysis

Antibiotic susceptibility data were analyzed using WHONET 5.6. Chi-square tests were used to determine between-group differences and for trend analysis. All analyses were performed in SPSS 23.0 (SPSS Inc., Chicago, IL, USA). Significance was set at *p* < 0.05.

## Results

### Pathogen distribution in orthopedics patients

Among the 1392 pathogen strains isolated from patients (Fig. 1a), 399 (28.7%) were Gram-positive, 982 (70.5%) were Gram-negative, and 11 (0.8%) were fungi. Additionally, 547 strains (39.3%) were recovered from wound secretions; 374 (26.9%) from incisional secretions; 223 (16.0%) from urine; 157 (11.3%) from sputum; 61 (4.4%) from blood; 14 (1%) from joint fluids; and 16 (1.1%) from other specimens (Fig. 1b). During the 6-year period (Table 1), *E. coli* (14.7%, 204/1392) was the most common pathogen responsible for nosocomial infection, followed by *Enterobacter cloacae* (13.9%, 193), *S. aureus* (11.3%, 157), *Pseudomonas aeruginosa* (9.8%, 136), *Acinetobacter baumannii* (9.6%, 134), *Staphylococcus epidermidis* (6.5%, 90), *Klebsiella pneumoniae* (4.6%, 64), and *Enterococcus faecalis* (3.2%, 44).

**Fig. 1:** **a** Classification of pathogenic bacteria. **b** Source of specimens

**Table 1:** Strains isolated from patients with HAIs from 2012 to 2017

	2012	2013	2014	2015	2016	2017	Total
*E. coli*	38 (15.1%)	39 (17.8%)	36 (18.3%)	40 (15%)	29 (11.8%)	22 (10.4%)	204
*E. cloacae*	40 (15.9%)	33 (15.1%)	18 (9.1%)	28 (10.5%)	34 (13.8%)	40 (18.9%)	193
*S. aureus*	28 (11.1%)	28 (12.9%)	33 (16.8%)	28 (10.5%)	24 (9.8%)	16 (7.5%)	157
*P. aeruginosa*	28 (11.1%)	17 (7.8%)	23 (11.7%)	26 (9.8%)	22 (8.9%)	20 (9.4%)	136
*A. baumannii*	22 (8.7%)	24 (11%)	16 (8.1%)	24 (9.0%)	24 (9.8%)	24 (11.3%)	134
*S. epidermidis*	16 (6.3%)	14 (6.4%)	13 (6.6%)	15 (5.6%)	16 (6.5%)	16 (7.5%)	90
*K. pneumoniae*	12 (4.8%)	10 (4.6%)	9 (4.6%)	13 (4.9%)	10 (4.1%)	10 (4.7%)	64
*E. faecalis*	8 (3.2%)	6 (2.7%)	7 (3.6%)	9 (3.4%)	8 (3.3%)	6 (2.8%)	44
*The others*	60	48	42	83	79	58	370
Total	252	219	197	266	246	212	1392

### Drug resistance rate of major pathogens

The dominant Gram-negative and Gram-positive bacteria causing nosocomial infections were respectively *E. coli* and *S. aureus*. Almost all *S. aureus* strains were resistant to penicillin (90.9–100%) and ampicillin (100%); over half were resistant to oxacillin, ceftriaxone, and erythromycin (Table 2). Fewer strains were resistant to levofloxacin, ciprofloxacin, and cotrimoxazole. None was resistant to nitrofurantoin, linezolid, and vancomycin. Trend analysis showed that *S. aureus* resistance to tetracycline significantly decreased (53.8% in 2012 and 37.5% in 2017, *p* = 0.026), whereas resistance to amoxicillin-clavulanic acid rose (20% in 2012 and 50% in 2017, *p* = 0.035).

**Table 2:** Trend of drug resistance rate of *S*. *aureus* in orthopedics from 2012 to 2017

Antibiotics	Drug resistance rate [%(strains/strains)]						Value	
	2012	2013	2014	2015	2016	2017	*χ*^2^	*p*
Penicillin	100.0 (20/20)	100.0 (16/16)	100.0 (20/20)	90.9 (20/22)	100.0 (20/20)	100.0 (14/14)	---	---
Oxacillin	50.0 (12/24)	39.1 (9/23)	53.1 (17/32)	50.0 (13/26)	60.9 (14/23)	75.0 (12/16)	5.632	0.344
Amoxicillin-clavulanic acid	20.0 (4/20)	37.5 (6/16)	59.1 (13/22)	60.9 (14/23)	66.7 (12/18)	50.0 (8/16)	12.006	0.035
Ceftriaxone	…	50.0 (8/16)	52.4 (11/21)	47.8 (11/23)	73.7 (14/19)	75.0 (12/16)	5.488	0.241
Levofloxacin	25.0 (6/24)	18.2 (4/22)	21.9 (7/32)	14.8 (4/27)	25.0 (6/24)	25.0 (4/16)	1.330	0.932
Tetracycline	53.8 (14/26)	27.3 (6/22)	42.3 (11/26)	11.5 (3/26)	25.0 (6/24)	37.5 (6/16)	12.740	0.026
Ciprofloxacin	33.3 (8/24)	18.2 (4/22)	33.3 (11/33)	14.8 (4/27)	25.0 (6/24)	25.0 (4/16)	4.104	0.535
Gentamicin	41.2 (12/26)	20.0 (4/20)	25.0 (8/32)	16.7 (4/26)	45.8 (11/24)	37.5 (6/16)	10.161	0.071
Cotrimoxazole	21.4 (6/28)	16.0 (4/25)	12.1 (4/33)	11.1 (3/27)	8.3 (2/24)	12.5 (2/16)	2.270	0.829
Ampicillin	100.0 (20/20)	100.0 (17/17)	100.0 (23/23)	100.0 (21/21)	100.0 (20/20)	100.0 (12/12)	---	---
Erythromycin	83.3 (20/24)	50.0 (11/22)	75.0 (24/32)	76.9 (20/26)	66.7 (16/24)	75.0 (12/16)	7.076	0.211
Nitrofurantoin	0.0 (0/14)	0.0 (0/6)	0.0 (0/6)	0.0 (0/5)	0.0 (0/6)	0.0 (0/7)	---	---
Linezolid	0.0 (0/26)	0.0 (0/22)	0.0 (0/30)	0.0 (0/25)	0.0 (0/24)	0.0 (0/16)	---	---
Vancomycin	0.0 (0/12)	0.0 (0/22)	0.0 (0/26)	0.0 (0/26)	0.0 (0/24)	0.0 (0/16)	---	---

…: Means that antibiotic was not tested or the results were not available in that year

---: Means that the chi-square value cannot be calculated

Most *E. coli* strains (81.8–93.3%) were resistant to ampicillin (Table 3). Approximately half were resistant to levofloxacin, ciprofloxacin, gentamicin, and cotrimoxazole (Table 3). Less than 20% of strains were resistant to amikacin, cefoperazone-sulbactam, meropenem, imipenem, and piperacillin-tazobactam. We observed a significant decrease in *E. coli* resistance to cotrimoxazole over time (47.1% in 2012 and 36.4% in 2017, *p* = 0.042), whereas resistance to imipenem and piperacillin-tazobactam significantly increased.

**Table 3:** Trend of drug resistance rate of *E. coli* in orthopedics from 2012 to 2017

Antibiotics	Drug resistance rate [%(strains/strains)]						Value	
	2012	2013	2014	2015	2016	2017	*χ*^2^	*p*
Amikacin	16.7 (4/24)	8.8 (3/34)	3.0 (1/33)	10.5 (4/38)	10.7 (3/28)	0.0 (0/22)	5.651	0.311
Ceftazidime	28.6 (8/28)	51.5 (17/33)	58.1 (18/31)	45.9 (17/37)	42.9 (12/28)	45.5 (10/22)	5.760	0.330
Cefepime	26.7 (8/30)	33.3 (11/33)	48.5 (16/33)	48.6 (18/37)	42.9 (9/21)	…	5.033	0.284
Cefoxitin	…	…	25.0 (4/16)	12.5 (3/24)	24.0 (6/25)	10.0 (2/20)	2.205	0.488
Levofloxacin	53.3 (16/30)	51.5 (17/33)	51.5 (17/33)	36.8 (14/38)	60.7 (17/28)	63.6 (14/22)	5.558	0.352
Tobramycin	27.3 (6/22)	23.5 (8/34)	25.0 (6/24)	28.6 (10/35)	28.6 (8/28)	36.4 (8/22)	1.226	0.942
Cefperazone-sulbactam	7.1 (2/28)	3.0 (1/33)	8.3 (2/24)	0.0 (0/17)	10.5 (2/19)	10.0 (2/20)	3.139	0.709
Ciprofloxacin	53.3 (16/30)	51.5 (17/33)	57.6 (19/33)	39.5 (15/38)	42.1 (16/28)	45.5 (10/22)	3.337	0.648
Gentamicin	60.0 (18/30)	54.5 (18/33)	51.5 (17/33)	34.2 (13/38)	46.4 (13/28)	45.5 (10/22)	5.427	0.366
Cotrimoxazole	47.1 (16/34)	67.6 (23/34)	75.8 (25/33)	57.1 (20/35)	57.1 (16/28)	36.4 (8/22)	11.493	0.042
Meropenem	0.0 (0/28)	3.3 (1/30)	6.1 (2/33)	8.3 (2/24)	19.2 (5/26)	10.0 (2/20)	7.476	0.124
Imipenem	6.7 (2/30)	2.9 (1/34)	3.0 (1/33)	0.0 (0/38)	17.9 (5/28)	9.1 (2/22)	9.130	0.043
Ampicillin	93.3 (28/30)	97.0 (33/34)	93.8 (30/32)	91.9 (34/37)	92.9 (26/28)	81.8 (18/22)	4.108	0.530
Piperacillin-tazobactam	0.0 (0/30)	2.9 (1/34)	3.0 (1/33)	0.0 (0/38)	17.9 (5/28)	18.2 (4/22)	14.370	0.010

…: Means that antibiotic was not tested or the results were not available in that year

---: Means that the chi-square value cannot be calculated

### Frequency of multidrug-resistant strains

The proportion of MRSA isolates was 43.3% (range: 28.6–62.5%), and the proportion of ESBL-positive *E. coli* isolates was 74.2% (range: 63.6–79.5%) (Fig. 2).

**Fig. 2:** Frequency of methicillin-resistant *S. aureus* (MRSA) and extended-spectrum β-lactamase (ESBL)-producing *E. coli* in orthopedics patients from 2012 to 2017

### Risk factors linked to MDR bacteria

Open fractures(Gustillo III B and IIIC) and degenerative diseases were significantly correlated with MDR bacterial infections (*p* < 0.05) (Table 4). Elderly patients exhibited a trend of increased susceptibility to MDR bacterial infections, but this effect was not significant. Finally, history of smoking and alcohol, diabetes, hypertension, and sex were not risk factors for infection with MDR bacteria.

**Table 4:** Demographic and clinical characteristics of MDR bacteria

	MSSA (*n* = 89)	MRSA (*n* = 68)	*χ*^2^	*p*	ECO(ESBL−) (*n* = 53)	ECO(ESBL+) (*n* = 151)	*χ*^2^	*p*
**Age**			2.451	0.484			3.871	0.274
< 20	10	11			2	5		
20–39	14	15			3	23		
40–59	47	32			23	66		
≥ 60	18	10			25	57		
**Gender**			0.077	0.781			0.316	0.574
Male	65	51			28	73		
Female	24	17			25	78		
**Smoking (*n*, %)**	5 (5.6)	6 (8.8)	0.215	0.643	7 (13.2)	22 (14.6)	0.060	0.807
**Alcohol (*n*, %)**	7(7.9)	9(13.2)	1.215	0.270	6 (11.3)	13 (8.6)	0.096	0.757
**Diabetes (*n*, %)**	6 (6.7)	7 (10.3)	0.641	0.424	7 (13.2)	15 (9.9)	0.437	0.509
**Hypertension (*n*, %)**	7 (7.9)	6 (8.8)	0.047	0.829	12 (22.6)	26 (17.2)	0.761	0.383
**Disease entities**								
Open fracture								
Gustillo I	7	9	3.151	0.076	5	9	0.028	0.868
Gustillo II	7	8	2.283	0.131	4	9	0.000	1.000
Gustillo III A	3	5	1.637	0.201	3	8	0.000	1.000
Gustillo III B	1	5	4.178	0.041	1	3	0.069	0.793
Gustillo III C	1	6	5.666	0.017	1	2	0.332	0.564
Degenerative disease (*n*, %)	25 (28.1)	14 (20.6)	1.162	0.281	11 (20.8)	59 (39.1)	5.840	0.016

## Discussion

In our study, *E. coli* was the predominant pathogen, followed by *E. cloacae*, *S. aureus*, *P. aeruginosa*, and *A. baumannii* (9.6%), similar to several previous findings [15, 16]. However, a cross-sectional descriptive study found that *P. aeruginosa* was the predominant microorganism (36.17%) causing nosocomial infections in orthopedics, whereas *E*. *coli* was only the fourth most prominent (6.38%); *E. cloacae* and *S. aureus* were even rarer [17]. This apparent discrepancy is likely due to the different procedures and tissue samples. Sarker et al. [17] only surveyed pathogens isolated from incisional secretions, but here, we surveyed pathogens isolated from a much larger variety of samples. For example, *E. coli* and *S. aureus* were frequently found in non-incisional secretions, such as urine [18]. Another reason for the difference may be that the two hospitals have dissimilar disease entities. A third of the orthopedics patients in the hospital we investigated were in the trauma division, and a study carried in Sichuan province, China, found that Gram-negative bacilli were the most common isolates and that *S. aureus* was the most common Gram-positive bacterium in trauma patients [19]. Finally, social, economic, and environmental variations may also account for between-study differences in different countries [20, 21].

Among the most widespread bacteria worldwide, *E. coli* is a known cause of urinary tract and bloodstream infections [18, 22]. The antibiotic-resistance patterns of *E. coli* in this study corresponded to those in previous reports [16, 23, 24]. Taken together, the findings suggest that we should reduce the usage of antibiotics to which *E. coli* is highly resistant, such as ampicillin. Additionally, we also recommend restricted usage of third-generation cephalosporins, despite observing low resistance. Our study identified a high percentage of ESBL-producing *E. coli*, and third-generation cephalosporins are the main factors leading to the emergence and spread of these strains [25].

In the event of *E. coli* infection, we recommend cautious use of antibiotics to which the bacterium is less resistant (e.g., amikacin). Currently, many doctors use empirical antibiotics without waiting for sensitivity reports [26, 27]. Fortunately, an antibiotic with a rate of accumulated bacterial resistance below 15% should be safe for use in empiric therapy [28]. Nevertheless, during the course of our 6-year study, we observed a clear increase in resistance to imipenem and piperacillin-tazobactam. This outcome serves as a warning against excessive antibiotic prescription, even if the target bacteria are initially less resistant.

*Staphylococcus aureus* was the dominant Gram-positive bacteria causing nosocomial infections in our study, in line with previous reports [29–31]. Specifically, we found high proportions of MRSA. Previous studies have similarly identified penicillin-resistant *S. aureus* [32], and indeed, our study identified only two *S. aureus* strains that were sensitive to penicillin. Furthermore, all strains were resistant to ampicillin. Together, these results indicate the real danger of MDR *S. aureus*. We therefore strongly advise against the empiric use of both penicillins and ampicillins. In contrast, *S. aureus* was not resistant to nitrofurantoin, linezolid, or vancomycin, suggesting that they can be safely used in clinics [33]. However, a vancomycin-resistant *S. aureus* isolate was reported in 2002, and subsequently, 14 isolates have been found in the United States [34]. Therefore, the three antibiotics should only be used in severe infections that cannot be controlled by other antibiotics. Fluoroquinolones and cotrimoxazole may be preferable, as our data show that *S. aureus* strains are not resistant to them. If neither is available, tetracycline can be a viable alternative based on the observed sensitivity of *S. aureus* to this drug [8].

Importantly, our findings clearly demonstrated a major problem with antimicrobial resistance in the study hospital, corroborating worldwide trends. Given that MDR bacteria are now recognized as a major cause of nosocomial infections [35], hospitals must work to control their incidence rate. Here, 43.3% and 74.2% of the strains were MRSA isolates and ESBL-positive *E. coli*, respectively, similar to a previous study in China [24]. The similarity suggests that some demographic and clinical characteristics could increase the risks of MDR bacterial infections. Indeed, we showed that patients with open fractures(Gustillo III B and IIIC) are more susceptible to MRSA infections, consequently contributing to multiple complications [36]. Regular attempts by surgeons to control infection via antibiotics likely explains the increased MDR in bacteria.

We observed a significant link between ESBL-producing *E coli* infections and degenerative diseases, which mainly affect elderly patients. Previous studies have indicated that elderly patients are at high risk of nosocomial infections, especially from MDR bacteria [24, 37]. This age-related risk was somewhat supported in our study, although we did not identify a significant relationship between elderly patients and MDR bacterial infections. Finally, other potential risk factors like biological sex, recreational drug use, diabetes, and hypertension did not increase the likelihood of multidrug-resistant bacterial infections [38, 39].

However, our research had some limitations. First, we only analyzed the drug resistance of the major bacteria, and thus, our findings may not be fully representative of the drug resistance of the whole department. Second, we did not analyze the bacterial spectrum and drug resistance in different disease entities. Further studies are therefore required to address these issues.

## Conclusions

We found that *E coli* and *S. aureus* were, respectively, the dominant gram-negative and gram-positive bacteria responsible for nosocomial infections in orthopedics. Drug resistance patterns of these pathogens demonstrated that antimicrobial resistance remains a serious concern. Notably, doctors must be aware of the infection risk from MDR bacteria. Our results lead us to strongly advocate extensive and dynamic monitoring of MDR bacteria, along with cautious antibiotics use, to effectively control antimicrobial resistance in pathogens.

## Data Availability

Data are available from the corresponding author on reasonable request.

## Abbreviations

HAI: Hospital-acquired infections
ICU: Intensive care unit
MRSA: Methicillin-resistant *S. aureus*
ESBL: Extended-spectrum β-lactamase
MDR: Multidrug-resistant
